The article "Risk Analysis of Positive PD-L1 Expression and Clinicopathological Features and Survival Prognosis in Patients with Colorectal Cancer: Systematic Review and Meta-Analysis" was retracted in 2023. Reasons: unreliable results or conclusions; concerns about the data; concerns about the peer review; concerns about the citations.

# Risk Analysis of Positive PD-L1 Expression and Clinicopathological Features and Survival Prognosis in Patients with Colorectal Cancer: Systematic Review and Meta-Analysis

**DOI:** 10.1155/2022/8212486

**Published:** 2022-04-11

**Authors:** Maocai Tang, Ziling Zheng, Jingkun Shang, Shouru Zhang

**Affiliations:** Department of Gastrointestinal Surgery, Chongqing University Cancer Hospital, Chongqing 400044, China

## Abstract

In order to explore the significance of PD-L1 expression in the prognosis and clinicopathological characteristics of colorectal cancer (CRC), the PubMed, Embase, Web of Science, Cochrane Library, CNKI, and multisquare databases are systematically searched for the relevant relationship between PD-L1 expression and CRC prognosis. The search time is completed until June 2021. Literature is filtered and data extracted by inclusion exclusion criteria, and Meta-analysis is performed with Stata SE12.0 software. 16 documents are included, and a total of 1997 CRC patients are included. The results show that recurrence-free survival (RFS) [OR = 2.69, 95%CI (2.07,3.48), *P* < 0.00001, I^2^ = 0%, *Z* = 7.50), and disease-free survival (DFS) (OR = 3.71, 95% CI (2.32,5.93), *P* < 0.00001, I^2^ = 37%, *Z* = 5.48) and PD-L1 expression and tumor differentiation (OR = 4.00, 95%CI (2.97,5.38), *P* < 0.00001, I^2^ = 0%, *Z* = 9.11) and lymphatic action metastasis (OR = 2.69,95% CI (2.07,3.48), *P* < 0.00001, I^2^ = 0%, *Z* = 7.50) is significantly associated.PD-L1 expression in tumor tissue suggests a poor prognosis in colorectal cancer, and the predictive significance of PD-L1 expression and PD-L1 expression in tumor cells in tumor-infiltrating immune cells may be inconsistent.

## 1. Introduction

Colorectal cancer (CRC) is one of the leading causes of cancer-related deaths, and over 2.2 million new cases and 1.1 million patient deaths are expected by 2030 [1]. The early symptoms of CRC are not specific, and many patients miss the optimal treatment time, and the first diagnosis is already progressive. Around 50% of patients will end up in metastatic colorectal cancer *Cancer*, mCRC). Most mCRC patients lose the chance of radical surgery and have poor prognosis [2]. Standard chemotherapy regiments for mCRC include FOLFOX (oxaliplatin + fluorouracil + leucovorin), FOLFIRI (irinotican + fluorouracil + leucovorin) and XELOX, et al. With the development and application of monoclonal antibodies against vascular endothelial growth factor (VEGF) and epidermal growth factor receptor (EGFR), Standard chemotherapy combined with targeted therapy results in improved outcomes in patients with mCRC [3]. But overall, the prognosis of mCRC is still suboptimal [3]. In recent years, immune checkpoint blocking therapy has made important progress, and immune checkpoint blocking therapy targeting the PD-1/PD-L1 pathway has achieved remarkable efficacy in the treatment of human solid tumors such as malignant melanoma, non-small-cell lung cancer, renal cell cancer, lymphoma, and breast cancer [4].

The article "Risk Analysis of Positive PD-L1 Expression and Clinicopathological Features and Survival Prognosis in Patients with Colorectal Cancer: Systematic Review and Meta-Analysis" was retracted in 2023. Reasons: unreliable results or conclusions; concerns about the data; concerns about the peer review; concerns about the citations.

For CRC, the PD-1 inhibitors Pembrolizumab and Nivolumab have been recommended by the seventh edition of the NCCN guidelines as postline treatment of mismatch repair defects/microsatellite highly unstable (dMMR/MSI-H) molecular phenotypic mCRC [5]. However, CRC is a highly molecular heterogeneous disease, and patients with different molecular phenotypes may respond to immunotherapy in very different ways, and finding new predictors for the benefit population of targeted immunotherapy [6].

PD-L1, also known as CD274 or B7–H1, is the main ligand of PD-1 and is a negative immunoregulatory protein [7]. PD-L1 is often expressed in tumor cells, dendritic cells, macrophages, fibroblasts, and T cells. By upregulation of PD-L1 expression and binding with PD-1, tumor inhibits THE activation of T cells, limits the strength of autoimmunity, and weakens the monitoring role of the immune system on tumor cells, resulting in immune escape. This is related to tumor genesis and development, and is the potential cause of poor prognosis of malignant tumor. PD-L1 is a potential predictor of CRC. Currently, published studies have been controversial on the relationship between PD-L1 expression and the prognosis of CRC. The Programmed Death 1 Ligand 1 (PD-L1) is a ligand of the programmed death receptor 1 (Programmed Death 1, PD-1). PD-1 is a member of the B7 familial costimulatory molecules, usually located in activated T cells and also expressed on the surface of B cells and NK cells, PD-L1 is located on the tumor or immune cell surface, PD-1 as a kind of the immune checkpoint, can negatively regulate T cell immunity Epidemic, the inhibition of T cell hyperactivation. PD-1 interacts with PD-L1 to block the CD28 signaling pathway, thereby inhibiting T cell activation [8]. The combination promoted the formation of an immunosuppressive tumor microenvironment. Numerous studies have shown that PD-L1 plays an important role in malignant melanoma, renal cell carcinoma, non-small cell lung cancer, and head and neck squamous cell carcinoma, which is both an important indicator indicating poor prognosis and an important target for clinical drug studies [9, 10]. In 2020, the US Drug and Food Administration (Food and Drug Administration, FDA) approved pembrolizumab and nivolumab for the treatment of malignant melanoma and non-small cell lung cancer [11–13].

The article "Risk Analysis of Positive PD-L1 Expression and Clinicopathological Features and Survival Prognosis in Patients with Colorectal Cancer: Systematic Review and Meta-Analysis" was retracted in 2023. Reasons: unreliable results or conclusions; concerns about the data; concerns about the peer review; concerns about the citations.

In order to provide large sample data to explore the significance and value of PD-L1 as a predictive factor of CRC, this study combined published research data on PD-L1 expression and PROGNOSIS of CRC with the method of meta-analysis, and evaluated the prognostic significance of PD-L1 expression and related clinicopathological parameters in CRC.

## 2. Our Proposed Method

### 2.1. Literature Retrieval Strategy

The correlation between PD-L1 expression and CRC prognosis is screened by using Library, CNKI and Wanfang database. Retrieval time is completed in June 2020. Retrieve vocabulary:“Colorectal cancer,” “Colorectal tumor,” “Colorectal neoplasm,” “Colorectal carcinoma,” “Colon cancer,” “Rectal cancer,” “PD-L1,” “CD274,” “B7–H1,” “Prognosis,” as shown in Figure 1.

### 2.2. Literature Inclusion Criteria

(1) All included patients are pathologically diagnosed with colorectal cancer; (2) the specimens came from tumor tissue and the PD-L1 expression is detected by immunohistochemistry (immunohistochemistry, IHC); (3) provided survival data for analysis, such as the HR of OS, RFS or DFS and its 95% CI, exploring the relationship between PD-L1 expression and CRC prognosis and (or) related clinicopathological parameters; (4) the publication language included in the literature is limited to Chinese and English.

### 2.3. Data Fetch

Two researchers independently screened the literature and extracted the data according to the set criteria. In case of different views, group discussion can be conducted to resolve disputes, to reduce errors in data extraction and increase heterogeneity and affect the final results. Firstly, duplicate literature are removed, and then the title and abstract of the article are read to exclude literature that did not meet the requirements of this study. Finally, the full text is read and the studies that met the requirements of inclusion are carefully screened. The extracted data included: (1) basic information: first author, country, publication date, antibody type, follow-up time, PD-L1 positive rate and truncation value; (2) relevant clinical medical records: sex ratio and number of cases in each study; (3) pathological characteristics: tumor size, TNM stage, depth of invasion, degree of tumor differentiation, vascular invasion, lymph node metastasis, chemotherapy, MSI status, KRAS mutation, et al. (4) survival prognosis data: OS (Overall survival), RFS (relapsefree survival) and DFS (disease-free survival) HR and 95%CI.

### 2.4. Literature Quality Evaluation and Bias Analysis

The Newcastle–Ottawa Scale (NOS) is used to assess the quality of the included literature, which included three parameters: selection, comparability and outcome assessment with a total score of 9 and a literature score above 6 is considered as high quality. Quality assessment is conducted independently by 2 researchers with group discussion addressing scoring inconsistencies and determining final inclusion in the literature after excluding low-quality literature.  Figure 2 is literature quality evaluation chart.  Figure 3 shows funnel plot of literature publication bias.

The article "Risk Analysis of Positive PD-L1 Expression and Clinicopathological Features and Survival Prognosis in Patients with Colorectal Cancer: Systematic Review and Meta-Analysis" was retracted in 2023. Reasons: unreliable results or conclusions; concerns about the data; concerns about the peer review; concerns about the citations.

### 2.5. Statistical Analysis

Risk ratio (HR) and 95% CI are used to evaluate the relationship between PD-L1 expression and COLORECTAL cancer OS, RFS, and DFS. Survival data are obtained directly from the literature. Odds ratios (OR) and their 95% CI are used to assess the association between PD-L1 expression and clinicopathological features associated with colorectal cancer. Statistically significant heterogeneity is defined *T* test *P* < 0.1 or I2 > 50%. If heterogeneity is observed, we use a random-effects model to reduce the impact of heterogeneity on the results; otherwise, we use a fixed-effects model. Egger's and Begg's tests are used to evaluate publication bias. All statistical analyses are performed using Stata SE12.0 software.

## 3. The Experimental Result

### 3.1. General Characteristics of the Included Literature

In this study, Pubmed, Cochrane, Web of Knowledge, Embase, CBM, CNKI, CECDB, and CQVIP are searched. A total of relevant literature are retrieved in the initial screening. Repeated publications and RCTs are excluded by reading titles and abstracts, and 16 literature are left. 16 full papers are reviewed, different reports of the same clinical study and literature inconsistent with the content of this study are excluded, and references of relevant literature are searched to prevent literature omission. Finally, a total of 16 RCTs are included in the study. All the retrieval and screening processes are completed by two evaluators independently, and any different opinions are unified through internal discussion, as shown in Table 1.

### 3.2. Correlation Analysis between PD-L1 Expression and OS in Colorectal Cancer

Among the 4 RCTs literature included in correlation analysis between PD-L1 expression and OS in colorectal cancer, heterogeneity test is carried out and it is found that the heterogeneity of the selected studies is small, so meta-analysis with fixed models could be performed. Meta-analysis results showed that the rhombus and vertical lines did not intersect in the forest plot of correlation analysis between PD-L1 expression and OS for 4 included literature, so there is a statistical difference in incidence of PD-L1 expression and OS between the treatment group and the control group [OR = 2.87, 95% CI (2.18,3.78), *P* < 0.00001, I2 = 76%, *Z* = 7.48].  Figure 4 displays Meta-analysis of PD-L1 expression and OS in colorectal cancer between two groups.

The article "Risk Analysis of Positive PD-L1 Expression and Clinicopathological Features and Survival Prognosis in Patients with Colorectal Cancer: Systematic Review and Meta-Analysis" was retracted in 2023. Reasons: unreliable results or conclusions; concerns about the data; concerns about the peer review; concerns about the citations.

### 3.3. Correlation Analysis between PD-L1 Expression and RFS in Colorectal Cancer

Among the 4 RCTs literature included in correlation analysis between PD-L1 expression and RFS in colorectal cancer, heterogeneity test is carried out and it is found that the heterogeneity of the selected studies is small, so meta-analysis with fixed models could be performed. Meta-analysis results showed that the rhombus and vertical lines did not intersect in the forest plot of correlation analysis between PD-L1 expression and RFS for 4 included literature, so there is a statistical difference in incidence of PD-L1 expression and RFS between the treatment group and the control group (OR = 2.69, 95% CI (2.07,3.48), *P* < 0.00001, I2 = 0%, *Z* = 7.50).  Figure 5 shows meta-analysis of PD-L1 expression and RFS in colorectal cancer between two groups.

### 3.4. Correlation Analysis between PD-L1 Expression and DFS in Colorectal Cancer

Among the 4 RCTs literature included in correlation analysis between PD-L1 expression and DFS in colorectal cancer, heterogeneity test is carried out and it is found that the heterogeneity of the selected studies is small, so meta-analysis with fixed models could be performed. Meta-analysis results showed that the rhombus and vertical lines did not intersect in the forest plot of correlation analysis between PD-L1 expression and DFS for 4 included literature, so there is a statistical difference in incidence of PD-L1 expression and DFS between the treatment group and the control group [OR = 3.71, 95% CI (2.32,5.93), *P* < 0.00001, I2 = 37%, *Z* = 5.48].  Figure 6 displays Meta-analysis of PD-L1 expression and DFS in colorectal cancer between two groups.

### 3.5. Correlation Analysis between PD-L1 Expression and Tumor Differentiation in Colorectal Cancer

Among the 4 RCTs literature included in correlation analysis between PD-L1 expression and tumor differentiation in colorectal cancer, heterogeneity test is carried out and it is found that the heterogeneity of the selected studies is small, so meta-analysis with fixed models could be performed. Meta-analysis results showed that the rhombus and vertical lines did not intersect in the forest plot of correlation analysis between PD-L1 expression and tumor differentiation for 4 included literature, so there is a statistical difference in incidence of PD-L1 expression and tumor differentiation between the treatment group and the control group (OR = 4.00, 95% CI (2.97,5.38), *P* < 0.00001, I2 = 0%, *Z* = 9.11).  Figure 7 shows meta-analysis of PD-L1 expression and tumor differentiation in colorectal cancer between two groups.

The article "Risk Analysis of Positive PD-L1 Expression and Clinicopathological Features and Survival Prognosis in Patients with Colorectal Cancer: Systematic Review and Meta-Analysis" was retracted in 2023. Reasons: unreliable results or conclusions; concerns about the data; concerns about the peer review; concerns about the citations.

### 3.6. Correlation Analysis between PD-L1 Expression and Lymph Node Metastasis in Colorectal Cancer

Among the 4 RCTs literature included in correlation analysis between PD-L1 expression and lymph node metastasis in colorectal cancer, heterogeneity test is carried out and it is found that the heterogeneity of the selected studies is small, so meta-analysis with fixed models could be performed. Meta-analysis results showed that the rhombus and vertical lines did not intersect in the forest plot of correlation analysis between PD-L1 expression and lymph node metastasis for 4 included literature, so there is a statistical difference in incidence of PD-L1 expression and lymph node metastasis between the treatment group and the control group (OR = 2.69, 95% CI (2.07, 3.48), *P* < 0.00001, I2 = 0%, *Z* = 7.50].  Figure 8 is meta-analysis of PD-L1 expression and lymph node metastasis in colorectal cancer between two groups.

## 4. Result Discussion

Inhibitory receptor expression can activate the activity of costimulators, restrict the migration and proliferation of T cells and the release of cytotoxic mediators, so as to prevent excessive autoimmune, inflammatory response and avoid tissue damage, which is an immune protection mechanism of the human body. However, tumors enhance the immunosuppressive effects in the tumor microenvironment by up-regulating the inhibitory receptor expression, causing effector T cell failure and limiting the antitumor immune responses triggered by CD4+ and CD8+ T cells, which may ultimately lead to immune escape or tolerance. PD-L1, one of the inhibitory receptors, has been shown to be selectively expressed at tumor sites, a feature that enables 'tumor-targeted' immunomodulation. Immunotherapy targeting the PD-1/PD-L1 transduction pathway can prevent PD-1 from binding to PD-L1, release the function of T cells, restore the normal immune response, and rerecognize and attack tumor cells to achieve antitumor effects. Upregulation of PD-L1 expression is an important way for tumor to escape immune attack and then spread, relapse and metastasis, which may be associated with poor prognosis of tumor. However, existing studies have shown that the prognostic significance of PD-L1 expression in tumor tissues for colorectal cancer is still controversial. Therefore, we conducted a meta-analysis to explore the feasibility of using PD-L1 expression to predict the prognosis of CRC.

Although there has been a meta-analysis on the relationship between PD-L1 and CRC prognosis, the number of articles included, the analysis model and the selection of effect size remain to be discussed. In the meta-analysis on the relationship between PD-L1 and prognosis of human solid tumors published by Temraz S et al in 2019, it is shown that in the CRC subgroup, PD-L1 expression is related to the decline of 5-year OS. Since OR is used to evaluate tumor survival indicators instead of HR and only 2 studies are included, this may increase the bias of the study. In the other three relevant meta-analyses, there is no statistically significant association between PD-L1 expression and CRC prognosis. Since CRC is not a targeted study, the number of relevant included studies is small.

The article "Risk Analysis of Positive PD-L1 Expression and Clinicopathological Features and Survival Prognosis in Patients with Colorectal Cancer: Systematic Review and Meta-Analysis" was retracted in 2023. Reasons: unreliable results or conclusions; concerns about the data; concerns about the peer review; concerns about the citations.

The prognostic analysis results of this study showed that PD-L1 expression is associated with the decline of OS and RFS. Analysis of relevant clinicopathological parameters showed that PD-L1 expression level is associated with tumor differentiation and lymph node metastasis, and poor tumor differentiation and lymph node metastasis are risk factors for poor prognosis of CRC. These evidences support that positive PD-L1 expression is associated with shorter SURVIVAL of CRC and can be used as a prognostic predictor of CRC. The results of subgroup analysis showed that pD-L1 expression, polyclonal antibody and univariate analysis subgroup are correlated with the decrease of OS, and heterogeneity significantly decreased in polyclonal antibody and univariate analysis subgroup, suggesting that antibody type and HR assessment type may be the main sources of heterogeneity in the correlation analysis between PD-L1 expression and OS. Moreover, according to the results of subgroup analysis, PD-L1 expression in tumor cells and tumor-infiltrating immune cells is not consistent with OS and RFS, and only the former is statistically significant associated with adverse OS and RFS.

Indeed, in tumor tissues, PD-L1 can be expressed as in tumor cells and tumor-infiltrating immune cells (tumor-infiltrating immune cells, TILs). The production of TILs is an adaptive immune response, and its role in controlling human tumor growth and recurrence is controversial. It has been shown that TILs can promote tumor, of immune escape and metastasis. Furthermore, TILs, although proliferating and clearing tumor cells in vitro, in vivo, due to the tumor microenvironment. The presence of an immunosuppressive microenvironment formed by the upregulation of immune checkpoint molecules makes it difficult for T cells to exert their role. The analysis results of the present study show an inconsistency in the effect of PD-L1 expression in tumor cells and TILs on CRC prognosis, but are limited to fewer included studies on TILs, the results should be treated with caution and more well-designed cohort studies are needed to demonstrate the effect of PD-L1 expression in tumor-infiltrating immune cells on CRC prognosis.

The article "Risk Analysis of Positive PD-L1 Expression and Clinicopathological Features and Survival Prognosis in Patients with Colorectal Cancer: Systematic Review and Meta-Analysis" was retracted in 2023. Reasons: unreliable results or conclusions; concerns about the data; concerns about the peer review; concerns about the citations.

Compared with previous Meta-analysis, this study has the following advantages: (1) the included study and sample size increased the test efficiency of Meta-analysis; (2) explored the impact of PD-L1 expression on CRC prognosis in tumor cells and tumor-infiltrating immune cells; (3) the data are directly given by the included literature rather than from survival curves, reducing the error; (4) the sensitivity analysis proved the stability of the results. These features increase the credibility of the results of this meta-analysis.

## 5. Conclusion

PD-L1 expression in tumor tissues is associated with the shorter OS and RFS of CRC, tumor differentiation, and lymph node metastasis, and the predictive significance of PD-L1 expression in tumor cells and tumor-infiltrating immune cells on the prognosis of CRC may be inconsistent.

This paper has some limitations: (1) the types of antibodies used for immunohistochemistry are different, and the cut-off value (cut-off value) criteria for PD-L1 positive test are varied. No subgroup analysis of the cut-off value is the defect of this article, it may increase research bias; (2) CRC with different molecular phenotypes respond differently to immunotherapy. This meta-analysis failed to perform subgroup analysis due to the lack of support for different molecular phenotypes.

## Figures and Tables

**Figure 1:** Flow chart of the literature screening.

**Figure 2:** Literature quality evaluation chart. (a) Risk of bias graph. (b) Risk of bias summary.

**Figure 3:** Funnel plot of literature publication bias.

**Figure 4:** Meta-analysis of PD-L1 expression and OS in colorectal cancer between two groups.

**Figure 5:** Meta-analysis of PD-L1 expression and RFS in colorectal cancer between two groups.

**Figure 6:** Meta-analysis of PD-L1 expression and DFS in colorectal cancer between two groups.

**Figure 7:** Meta-analysis of PD-L1 expression and tumor differentiation in colorectal cancer between two groups.

**Figure 8:** Meta-analysis of PD-L1 expression and lymph node metastasis in colorectal cancer between two groups.

**Table 1:** Basic clinical features of 16 literature are included in our study.

Study	Age	Gender (Man)	Experimental group (N)	Control group (N)	NOS score	Research type	*P*
Brahmer JR 2012	63.71 ± 2.2	41.25	18/75	11/75	8	RCT	<0.05
Topalian SL 2012	55.65 ± 3.4	69.12	211/296	112/296	7	RCT	<0.05
O'Neil BH 2017	63.12 ± 4.5	45.72	33/137	12/137	8	RCT	<0.05
Chen EX 2020	62.15 ± 4.5	44.12	121/180	59/180	8	RCT	<0.05
Van dijk N 2020	62.85 ± 1.4	51.89	12/24	9/24	8	RCT	<0.05
Ott PA 2017	54.36 ± 1.2	63.45	32/43	11/43	7	RCT	<0.05
Kawazoe a 2020	52.62 ± 2.2	78.10	44/55	21/55	9	RCT	<0.05
Limagne E 2016	62.61 ± 3.0	48.75	15/25	6/20	9	RCT	<0.05
Hellmann MD 2019	47.25 ± 4.5	59.23	76/152	56/152	7	RCT	<0.05
Li J 2021	48.22 ± 5.2	56.22	29/65	18/65	8	RCT	<0.05
Lonardi S 2021	61.35 ± 1.1	53.16	23/30	18/27	8	RCT	<0.05
Kim JH 2020	61.25 ± 1.0	66.34	16/33	13/33	8	RCT	<0.05
Lau D 2020	58.51 ± 1.6	48.34	216/402	113/402	9	RCT	<0.05
Taylor K 2020	66.34 ± 1.5	53.12	19/28	9/28	9	RCT	<0.05
Levy A 2016	67.45 ± 3.6	67.12	6/10	4/10	7	RCT	<0.05
Shamseddine A 2020	63.65 ± 2.2	54.31	31/44	13/44	8	RCT	<0.05

The article "Risk Analysis of Positive PD-L1 Expression and Clinicopathological Features and Survival Prognosis in Patients with Colorectal Cancer: Systematic Review and Meta-Analysis" was retracted in 2023. Reasons: unreliable results or conclusions; concerns about the data; concerns about the peer review; concerns about the citations.

## Data Availability

The simulation experiment data used to support the findings of this study are available from the corresponding author upon request.

## References

[1] Franke A. J., Skelton W. P., Starr J. S. (2019). Immunotherapy for colorectal cancer: a review of current and novel therapeutic approaches. *Journal of the National Cancer Institute: Journal of the National Cancer Institute*.

[2] Picard E., Verschoor C. P., Ma G. W., Pawelec G. (2020). Relationships between immune landscapes, genetic subtypes and responses to immunotherapy in colorectal cancer. *Frontiers in Immunology*.

[3] Ijsselsteijn M. E., Sanz-Pamplona R., Hermitte F., de Miranda N. F. C. C. (2019). Colorectal cancer: a paradigmatic model for cancer immunology and immunotherapy. *Molecular Aspects of Medicine*.

[4] Kang H., Kiess A., Chung C. H. (2015). Emerging biomarkers in head and neck cancer in the era of genomics. *Nature Reviews Clinical Oncology*.

[5] Piawah S., Venook A. P. (2019). Targeted therapy for colorectal cancer metastases: a review of current methods of molecularly targeted therapy and the use of tumor biomarkers in the treatment of metastatic colorectal cancer. *Cancer*.

[6] Wrobel P., Ahmed S. (2019). Current status of immunotherapy in metastatic colorectal cancer. *International Journal of Colorectal Disease*.

[7] Song W., Tiruthani K., Wang Y. (2018). Trapping of lipopolysaccharide to promote immunotherapy against colorectal cancer and attenuate liver metastasis. *Advanced Materials*.

[8] Brahmer J. R., Tykodi S. S., Chow L. Q. M. (2012). Safety and activity of anti-PD-L1 antibody in patients with advanced cancer. *New England Journal of Medicine*.

[9] Topalian S. L., Hodi F. S., Brahmer J. R. (2012). Safety, activity, and immune correlates of anti-PD-1 antibody in cancer. *New England Journal of Medicine*.

[10] O’Neil B. H., Wallmark J. M., Lorente D. (2017). Safety and antitumor activity of the anti–PD-1 antibody pembrolizumab in patients with advanced colorectal carcinoma. *PLoS One*.

[11] Yan J., Zheng X., You W., He W., Xu G.-K. (2022). A bionic-homodimerization strategy for optimizing modulators of protein-protein interactions: from statistical mechanics theory to potential clinical translation. *Advanced Science*.

The article "Risk Analysis of Positive PD-L1 Expression and Clinicopathological Features and Survival Prognosis in Patients with Colorectal Cancer: Systematic Review and Meta-Analysis" was retracted in 2023. Reasons: unreliable results or conclusions; concerns about the data; concerns about the peer review; concerns about the citations.

[12] Jin K., Yan Y., Chen M. (2022). Multimodal deep learning with feature level fusion for identification of choroidal neovascularization activity in age‐related macular degeneration. *Acta Ophthalmologica*.

[13] Yan J., Yao Y., Yan S., Gao R., Lu W., He W. (2020). Chiral protein supraparticles for tumor suppression and synergistic immunotherapy: an enabling strategy for bioactive supramolecular chirality construction. *Nano Letters*.

